# Using the Improved SSD Algorithm to Motion Target Detection and Tracking

**DOI:** 10.1155/2022/1886964

**Published:** 2022-05-14

**Authors:** Yongjiang Yan

**Affiliations:** Xi'an Medical University, Xi'an City, Shaanxi 710021, China

## Abstract

Computer vision-based motion target detection and tracking, which is widely used in video surveillance, human-computer interaction, range interpretation, and other fields, is one of the current research hotspots in the field of computer vision. In engineering scenarios, the two are inseparable and need to work together to accomplish specific tasks. The related research is progressing rapidly, but there is still room for improving its timeliness, accuracy, and automation. In this paper, we summarize and classify some classical target detection methods, analyze the basic principles of convolutional neural networks, and analyze the classical detection algorithms based on region suggestion and deep regression networks. After that, we improve the SSD algorithm for the shortage of low-level feature convolution layers, which has insufficient feature extraction and leads to poor detection of small targets. For the motion target tracking problem, this paper studies the motion target tracking method based on support vector machine and proposes the tracking method of support vector regression and the corresponding online support vector regression solution method based on the analysis of support vector tracking method and structural support vector tracking method. In this paper, we propose a tracking method that fuses structural support vector machines and correlation filtering. The structure is based on the idea of Inception, which adds and replaces some feature convolution layers of the original network while maintaining the original lightweight backbone. The final experiments on the VOC data set demonstrate that the improved algorithm improves the average detection accuracy by 2.6% compared to the original algorithm and basically maintains the real-time speed as well. Experimental simulations on a subset of VOC data (human set) show a significant improvement in AP values and more effective and reliable detection tracking of moving targets. The stability and accuracy of motion target detection and tracking are improved by setting parameters, such as confidence level; the effectiveness and continuity of detection and tracking are judged by setting the interframe centroid distance.

## 1. Introduction

Target detection is a research hotspot in the field of computer vision and digital imaging, which is widely used in many fields, such as supporting robot navigation, intelligent video analysis, industrial production inspection, and so on [1]. Through the development of digital computers, which affect all aspects of people's production life, various specific tasks can be completed efficiently and quickly, reducing expenses while improving efficiency. In the good state of development of digital computer technology, on the one hand, digital computers can quickly deal with numerical calculations; on the other hand, it is more likely to improve the objective shortcomings of human vision itself, using computers to effectively process visual information [2]. The development of digital computer technology and the discipline of computer vision are promoting each other's development state, forming a win-win situation [3]. The purpose of computer vision research is to enable computers to play a perceptual effect on objective information that does exist in real-world physical objects, for example, perceiving shape, location, color, and movement, and can describe, classify, understand, and store that physical object, making this technology one of the popular research topics today. Target detection technology has universal application in many aspects, such as digital image discrimination, motion pedestrian detection, multiscene target analysis, and so on [4]. Improving the speed and accuracy of target detection has strong engineering value and significance, and related research has been carried out at home and abroad around this aspect, and the research results have been applied to engineering projects with certain achievements [5]. Particularly in recent years, the development of artificial intelligence and deep learning has brought new power to the research work of target detection and tracking recognition [6]. Motion target detection and tracking is a video analysis technology, and the research application of target tracking methods in video is one of the important branches of computer vision discipline, which is increasingly widely used in national science and defense construction, aerospace field, medical and health care, and other diverse people and welfare fields.

At this stage, the video surveillance system as an important technology in public social security has received strong attention from the general public and will be applied, but the function of many existing video surveillance system is still parked in 24-hour manual monitoring, which requires a lot of time and effort to monitor the content of the surveillance video, or the need to analyze and understand the video content of the surveillance video, to get effective support for the alarm information, and to provide technical support for the task of alarm [7]. In the digital computer video intelligent monitoring system, the video surveillance system will first be processed to the original image information for noise preprocessing operations, and then the appropriate target detection algorithm is used to detect to determine the motion of the object in the video, and then use the appropriate target tracking algorithm within the surveillance video to track the motion of the target in real time [8]. In addition, it will also assist in the implementation of system functions according to the actual needs, such as the use in police surveillance, which will be responsible for a series of related tasks, such as early warning or alerting. At present, the main interface path commonly used to interact with computer is through keyboard and mouse. With the development of science and technology, in order to respond to the needs of all aspects of production and life, the current human-computer interaction mode has been improved, becoming more intelligent and life more convenient [9]. Through computer perception, we can collect the contactless video signal input by the user through the computer, analyze the processing operation of the video signal through the relevant theory under the background of computer vision, understand the user's posture and action form, and judge the user's meaning, so that the original mechanical computer can understand each other as much as possible like a friend and output the results of computer processing. Current research in the field of work that allows computers to recognize and analyze and understand human actions focuses on gesture analysis [10], expression understanding, action judgment, and other similar aspects in order for computers to form autonomous recognition and judgment of these human postures or actions. Similarly, the research in these aspects of technology is where breakthroughs in the development of robots are being made today. In addition, target detection and tracking technology has been applied and developed in fields such as automated agricultural production and medical image content reconstruction [11]. Target detection and tracking technology is the underlying technology of computer vision system, which is the key and basic link of various subsequent advanced processing [12].

The target detection and tracking technology has the necessary research value and profound application prospects. Due to the variable complexity of the real environment, there are still problems that need to be overcome in the actual engineering use of this technology. Range image measurement by visual means is a fundamental task in the missile development process, involving basic computer vision problems, such as detection and tracking of moving targets. The range image quality is greatly disturbed by the weather and imaging quality, the target frequently enters and leaves the field of view, and the multiscale performance of the target is obvious, all of which lead to the accuracy and efficiency of the traditional target detection, and tracking methods cannot adapt to the increasingly complex interpretation scenarios and the escalating data volume. Modern range optical image interpretation of real-time measurement image processing is based on post facto interpretation, which still stays at a more basic level of underlying vision, requiring a lot of manual intervention, mostly using human a priori, statistical information, and so on, to extract the target object color, texture, contour and geometric shape, and other underlying features, which are not robust enough to the target scene, resolution, and so on. Therefore, efficient and accurate target detection and tracking methods are crucial to the intelligence level of range interpretation. This topic focuses on efficient and accurate target detection and tracking methods and proposes certain solutions to the problems existing in traditional learning and deep learning methods for motion target detection and tracking, aiming to improve the timeliness and intelligence level of modern range optical tracking measurement. The studied motion target detection and tracking method is also applicable to other fields of computer vision, which has academic significance and engineering value.

## 2. Related Work

In the literature, a single Gaussian model and a background and threshold adaptive method are incorporated in the existing three-frame difference method, which effectively reduces the interference from background and noise and makes the target detection more complete [13]. In the literature, the hybrid Gaussian model is incorporated in the improved frame difference method to improve the deficiency of detecting the background as foreground in the detection process [14]. The literature takes advantage of the SIFT feature (scale-invariant feature transform) scale and rotation invariance can well meet the conditions of optical flow estimation, and the proposed algorithm with improved template update strategy has better detection accuracy for target partial occlusion [15]. The literature finds that the one-dimensional maximum entropy method obtains complete and accurate target information during detection, and the grayscale value with the maximum information entropy between the background and the target as the detection threshold can better achieve the detection of moving targets in complex backgrounds. The adaptive background modeling algorithm with Kalman filtering and dynamic region reconstruction is proposed in the literature to better solve the background model trailing defects caused by slow targets and also has good robustness to background noise. In order to improve the adaptability of the background extraction model in dynamic scenes, the literature combines visual saliency to determine the degree of pixel point ghosting in the background model and effectively improves the shortcomings of the Vibe (visual background extractor) algorithm by fusing the fuzzy criterion adaptive temporal subsampling factor. The literature [16] fused five-frame differential information and background edge detection information, and then morphologically found out more accurate detection results for the emergence of voids, shadows, and false edges.

The DPM (Deformable Part-based Model) algorithm proposed by Felzenszwalb in 2008 for generic target detection combines Histograms of Oriented Gradients (HOG) features, SVM (Support Vector Machine) classifier, and the algorithm combines the ideas of HOG (Histograms of Oriented Gradients) features, SVM (Support Vector Machine) classifier and sliding windows and was the winner of three PASCAL VOC target detection championships before the advent of deep neural networks. Later, with the influx of researchers and the improvement of large-scale databases, detection networks using convolutional neural networks developed rapidly. The representative ones include VGGNet [17] jointly proposed by Google and Oxford University Computer Vision Group, GoogLeNet proposed by Christian Szegedy and others, and ResNet proposed by Chinese scholars such as Kaiming He and others. At present, people generally classify the mainstream Anchor-based class target detection methods into single-shot and two-step approaches [18]. The most intuitive difference is that the former is faster, while the latter is better than the accuracy. In the two-stage approach, the candidate frames are used as samples for classification by convolutional neural networks, and the most studied are R-CNN (Regions with CNN Features) algorithm and the improved fast R-CNN and Faster R-CNN algorithms. In addition, the R-FCN (Region-based Fully Convolutional Network) algorithm proposed in 2016, the FPN (Feature Pyramid Networks) algorithm and the Mask R-CNN algorithm appeared in 2017, and so on [19].

The one-stage converts the target frame localization problem into a regression problem to be studied. The most influential one is the YOLO (You Only Look Once) algorithm based on OverFeat in 2015, followed by the YOLOv2 and YOLOv3 methods to address the shortcomings of each algorithm [20]. Another famous one is the SSD (Single-Shot MultiBox Detector) algorithm, which combines the idea of regression with the anchor box mechanism. There are also many improved methods such as DSSD (Deconvolutional Single-Shot Detector) algorithm, DSOD (Learning Deeply Supervised Object Detectors from Scratch) algorithm, and so on [21]. As the research continues, both types of algorithms have been greatly improved in terms of accuracy and speed, and this has accumulated experience and opened up directions for research in this field.

## 3. Neural Net-Based Motion Target Detection and Tracking

### 3.1. Motion Target Image Preprocessing

Digital image processing is simply the use of digital quantization techniques to correct images to improve their appearance, eliminate redundant information, and enhance and modify the image information needed for human observation. It mainly consists of image graying, binarization, denoising, and morphological operations. It is the basis of the research and the primary task of this paper. Grayscale image refers to an image that contains only luminance without color information. In contrast to color images, the “gray” color of a grayscale image means that the components of red, green, and blue have the same intensity in RGB space, so only one intensity value needs to be specified for each pixel, not three. Typically, grayscale intensities are stored as 8-bit integers, giving 256 possible different shades of gray from black to white. If these levels were evenly spaced apart, the difference between successive gray levels would be significantly better than the grayscale resolution of the human eye. In many applications of image processing, most of the information to be perceived is in the luminance component *Y* and not in the chromaticity components *U*, *V* or bC, Cr. Converting to grayscale images allows more complex operations to be performed in less time using smaller data. Grayscale processing can be used as a preprocessing step to build the foundation for later deeper operations, such as image segmentation, recognition, and analysis. The commonly used methods for grayscale are mean, maximum, and weighted average.

(1) The summation of R, G, and B components' luminance and then averaged to get a gray value is called the averaging method. That is,
  (1) $$\begin{array}{c} G_{\text{value}}=\frac{\left(\text{Red}+\text{Green}+\text{Blue}\right)}{3}. \end{array}$$
(2) Selecting the maximum value of luminance in R, G, and B components as the gray value of the image is called the maximum value method. That is,
  (2) $$\begin{array}{c} G_{\text{value}}=\frac{\text{Red}}{2}+\frac{\text{Green}}{3}+\frac{\text{Blue}}{2}. \end{array}$$
(3) Based on the sensitivity of the human visual system to color, the method of calculating the grayscale value by assigning different weights to the three components R, G, and B and then weighting the average is the weighted average method. That is,
  (3) $$\begin{array}{c} G_{\text{value}}=\frac{\text{Red}}{3}+\frac{\text{Green}}{5}+\frac{\text{Blue}}{3}. \end{array}$$

The binarization of images facilitates the extraction of valid information in the image and improves the recognition efficiency in the detection and tracking of targets. By binary image, we mean that all pixels in the image can only have grayscale values of 0 and 255, and the processed image is displayed as a black-and-white image. The process of binarization is done by artificially setting the appropriate threshold value and further taking out the gray value of each pixel point in the image to compare with the preset threshold value, the pixel with gray value greater than or equal to the set threshold value is determined to belong to a specific object and the gray value of that point is set to 255; the opposite is 0, indicating the background or the region where the exception object is located. The expressions are:

(4) $$\begin{array}{c} G_{\text{value}}\left(a,b\right)=\left\{\begin{array}{c} 0,q\left(x,y\right)<p,\\ 1,q\left(x,y\right)>p. \end{array}\right) \end{array}$$

Digital images are easily captured and transmitted by sensor devices or random signals from the external environment to generate noise that hinders subsequent analysis and understanding of the processing, which can interfere with the extraction of target motion image information and make the detection and tracking of the target in motion cause errors and affect the results. Therefore, it is very necessary to complete image denoising before implementing detection and tracking analysis of the target, which will directly improve the quality of subsequent motion information analysis. The main reason for noise in the image is that the transmission channel is contaminated by noise during transmission, which is generally classified as Gaussian noise, Rayleigh noise, gamma noise, exponential noise, and pretzel noise according to the characteristics of noise. The two most frequent noises in digital image processing are pretzel noise and Gaussian noise. Bright and dark dot noise from the image sensor, the transmitted channel, and the decoding process in black and white are the main causes of pretzel noise, and the cutting of the image is also very likely to trigger pretzel noise. High gray salt noise and low gray pepper noise usually appear at the same time, which is visualized as black-and-white noise on the image. Median filtering is the preferred method for dealing with pepper noise in general. The other is the most common Gaussian noise. Its probability density function obeys Gaussian distribution. Most of the time, Gaussian noise is easy to be generated in the process of image acquisition due to poor light or affected sensors. Generally, in order to reduce Gaussian noise, more spatial filters are used, as shown in Figure 1.

Median filtering, as a nonlinear smoothing technique, is essentially a statistical ranking filter. The principle is that for a specific point in an image, the current pixel point value is updated with the statistically ordered median of all pixels in the neighborhood surrounding the point. The two factors that affect its effectiveness are mainly the spatial extent of the neighborhood and the number of pixels. For certain types of random noise, it is able to eliminate or attenuate the high-frequency component of Fourier space, while also affecting the low-frequency component, and causes less blurring effect when compared to linear smoothing filters in reducing noise. The most typical application is for the elimination of pretzel noise, where median filtering has excellent noise reduction capabilities. Through computer sensing, the video signal is input through the computer and can be collected without contacting the computer user.

### 3.2. Neural Network Algorithm for Motion Target Detection

The interframe differencing method is one of the most frequently used methods for target detection and segmentation in static background. Since the environment in the field of view of the camera does not change much in a short period of time, the similarity of the background in the adjacent or similar frames is relatively high, so the region where the moving target is located can be obtained by taking the time domain difference of pixel grayscale between several adjacent or similar frames. If the pixel value of a point in the two frames for comparison is less than a predefined threshold, it is marked as a background pixel; otherwise, it is considered as a foreground pixel. The position of the moving target in the image frame can be extracted by using the marked foreground pixel points. Generally, a feature template can be formed by combining the edge features, linear features, center features, and diagonal features of Haar features. There are two types of rectangles within the feature template, white rectangle and black rectangle, and the value obtained by subtracting the total pixel sum of the white rectangle from the total pixel sum of the black rectangle within this template is the desired feature value of that image. The total pixel sum of any region in the image is obtained by the integration method of equation (5). The total pixel value *ii*(*i*, *j*) at position (*i*, *j*) in the image can be expressed as the sum of all pixel values in the direction of the upper left corner of point (*i*, *j*) on the image:

(5) $$\begin{array}{c} \text{Point}\left(i,j\right)=\frac{\sum q\left(i,j\right)}{G_{\text{value}}}. \end{array}$$

Generally speaking, when humans understand complex information, they first receive its manifested visual image information, such as color shades, brightness levels, edge shapes, corner features, straight curves, and so on; then, they proceed to receive its deeper texture features, geometric information, and so on. The principle of image processing by convolutional neural networks can be simply described as described in the above paragraph. Convolutional neural networks are basically composed of multiple convolutional layers connected in sequence, and each convolutional layer is set up with multiple convolutional kernels present. The convolutional kernels in each convolutional layer scan the entire processed image in a left-to-right, top-down order, and the data of the feature map is output. The different results obtained by different perceptual field operations in different layers are the information on different scales of the image. The convolutional layer and pooling layer are the key structures of convolutional neural networks. The convolutional layer consists of a set of convolutional units (convolutional kernels) that resemble filters, each of which extracts a specific feature, as shown in Figure 2.

The convolutional layer is the basic component of convolutional neural network and also a crucial part. In convolutional neural network, the convolutional layer is involved in feature extraction, and the quality of feature extraction directly affects the accuracy of later detection. The information of an image is embedded in all the pixel points of the image, and to extract the overall features of the image, all the pixel points of the image must be studied. In an image, the correlation between pixels in close proximity is high, and the correlation between pixel points in far distance is low:

(6) $$\begin{array}{c} I_{q-1}\left(x,y\right)=I_{q}\left(x,y\right)+I_{q+1}\left(x,y\right)+I_{q+2}\left(x,y\right)+...+I_{q+n}\left(x,y\right),\\ I_{q+1}\left(x,y\right)=I_{q}\left(x-1,y-1\right). \end{array}$$

Integrating the local information to get the whole information is a common way of image processing. Different sizes of convolution kernels affect the effect of feature extraction. An example of the basic convolution operation is shown in Figure 3. For an input matrix *M*, it is processed with a convolution kernel *F*. *F* is used to process the matrix by moving in fixed steps and performing dot product operations to obtain the final matrix:

(7) $$\begin{array}{c} I_{q}\left(x,y\right)=\alpha_{i}I_{q}\left(x-1,y-1\right)+\alpha_{i+1}I_{q}\left(x-1,y-1\right),\\ I_{q}\left(x,y\right)=\beta_{i}I_{q-1}\left(x,y\right)+\beta_{i+1}I_{q-1}\left(x,y\right). \end{array}$$

Then, the image of frame *t* + 1 obtained by Warp is

(8) $$\begin{array}{c} I_{q}\left(x,y\right)=\left\{\begin{array}{c} 0,q>1,\\ 1,q<1,\\ 2,q=1. \end{array}\right) \end{array}$$

### 3.3. Motion Target Tracking and Matching

In intelligent video analysis systems, motion target detection and tracking is a fundamental core link, and its performance is directly related to the accuracy of subsequent action recognition, behavior analysis, and other advanced semantic processing. Due to the complexity of the surveillance environment, the multiplicity, and concurrency of various interference factors, it is important to study motion target detection and tracking models with high accuracy, low time consumption, and guaranteed strong robustness. In intelligent surveillance, real-time trajectories can be formed and analyzed by real-time detection and tracking of pedestrians to obtain pedestrian-related events; in intelligent transportation, the direction of pedestrian activities can be predicted to effectively prevent traffic accidents; in pedestrian flow statistics, pedestrian flow monitoring and control can be implemented by analyzing pedestrian trajectories, and so on. In the actual motion target detection and tracking process, interference factors appear between video images, such as blurred picture quality caused by low pixel count of video acquisition, inconspicuous difference between background environment and the target itself, and different movements of the motion target itself leading to pose changes, obscured by other physical objects, and so on; all these related factors will cause detection difficulties in the target tracking process.

In this paper, we design the following scheme for the target detection and tracking task of moving pedestrians in video. The SSD network is used as a pedestrian target detection network, which can detect pedestrian targets of various sizes by using its principle of predictive recognition of categories at diverse scales. In the key frame image, which is the first frame in which the pedestrian appears in consecutive video frames, the SSD network extracts the deep semantic features in the model to detect the pedestrian for the first time and locks the detection target. Then, the SSD network continuously detects the moving pedestrian target in the current frame in each nonkey frame after the key frame, taking advantage of the high similarity between the moving pedestrian target in the front and back frames of the video. In case of false detection in one of the frames due to changes in the shape of the pedestrian target, changes in lighting, and other internal and external factors, the model structure and its parameters are immediately adjusted until the pedestrian target is successfully detected in every frame of the entire video sequence. The continuous detection of each frame in the continuous frame sequence forms the tracking effect of the pedestrian target. Since the output of the tracking model should be continuous, the model is updated in a timely manner based on the output when the model fails to track. After initializing the list of tracking points and initializing the center of mass of the target frame, the tracking points are traversed for all frames in the video, and the trajectory of the target is drawn by connecting all the traversed centers. Learning rate schedules attempt to change the learning rate during each update, and whatever adjustment process will be experienced, it is necessary to first fix the learning rate value settings.

The LSTM network is used to predict the trajectory of the moving pedestrian by learning the coordinate sequence of the trajectory of the moving pedestrian target, and the predicted trajectory is obtained based on the actual action trajectory of the moving pedestrian target. In this paper, the trajectory prediction of the moving pedestrian target is done by point-by-point prediction, as shown in Figure 4. In addition, since the movement of pedestrians is not abrupt, but has a certain regularity and continuity, and now pedestrian detection and monitoring has a significant effectiveness contribution in the field of automated driving, the estimation of the future range of action of pedestrians can provide a part of support to the operation judgment of automated driving and make a contribution in the field of automated driving. With the support of mathematical theory, the future trend range of the movement pedestrian target is calculated.

## 4. Experiments and Results Analysis

### 4.1. Data Enhancement

Data augmentation is an essential part of the training process for neural networks and is required in SSD networks as well. Among them, pixel content transformations and spatial geometry transformations of images are half of this data enhancement process. Pixel content transformation includes random change of image brightness, random change of contrast, chrominance, saturation, and random change of color channels. Spatial geometric transformations include random expansion, random crop, and random mirroring. In addition, there are coordinate transformation, resize and subtract means of image data. Among them, the detection and tracking of pedestrian targets is an important subfield in the field of motion target detection and tracking. Pedestrian target tracking is important in unmanned driving, intelligent surveillance, intelligent transportation, and so on.

In practice, it is found that SGD is simple, easy to implement, and can autonomously avoid undesirable local optimal points, and when it converges, the results found also have strong generality, so it can perform very well on data sets that it has not seen before but obey the same distribution. Since SGD updates the parameters of the model by selecting only a random amount of sample sets at a time to be trained by the network, the algorithm learns very quickly each time and can be updated online. The choice of the learning rate has a significant impact on the convergence of the optimizer, so it is challenging to choose a reasonable learning rate. If the learning rate of the network is too large, it will hinder the convergence of the optimizer; if the learning rate of the network is too small, it will cause the convergence of the optimizer to be too slow and image the overall running time of the network, as shown in Figure 5.

### 4.2. Evaluation Indicators

In this thesis, the average accuracy mean (AP) is used as the main performance evaluation metric for static target detection experiments. There are two methods to calculate the AP value; the first one is the 11-point calculation in 2017, which sets 11 thresholds for the recall rate, calculates the maximum accuracy rate in the case of greater than the threshold, and after obtaining 11 accuracy rates, the AP value is obtained by finding the average value; the second method is proposed in 2010, which calculates the area under the PR curve (the horizontal axis is the recall rate and the vertical axis is the accuracy) to obtain the AP value. VOC2007 defaults to IOU greater than 0.5 as TP, and the steps for calculating the average value of AP for multiple categories (i.e., MAP value) in this thesis are divided into the following steps: (1) calculate the precision P of a category in a single image; (2) loop all test set images and repeat the previous process to find the average value of all images P, which is the AP of that category; and (3) repeat the previous two processes for the remaining N-1 categories and this thesis uses the SSD network as the base model for experimental application, and after improvement, we obtain the double micro SSD network, which is applied to the actual life shooting scene video; with the base learning rate of 0.0001, the gradient descent method is random gradient descent method, and the number of samples for gradient descent and the batch size of batch training data is 32. The target object is detected, and the maximum score (score) detection category is framed and outputted for display. The performance of the detection results should not only consider the accuracy factor, but also the detection speed. The experimental results demonstrate that the experimental accuracy of the dual micro SSD network-based model on the VOC dataset reaches 0.927, and Figure 6 shows the performance comparison of various related models on the VOC dataset.

The SSD network and dual micro SSD both perform well in terms of accuracy, but the former has a slight advantage in detection time, and the improved dual micro SSD does not have a significant decrease in detection speed, but its accuracy is greatly improved, the Faster R-CNN network performs well in terms of accuracy, but its detection speed is relatively unsatisfactory, and YOLO is at a disadvantage in terms of detection accuracy. Video target tracking uses detection algorithms in key frames and optical flow in nonkey frames to assist in tracking, which results in a significantly slower tracking speed and a less than optimal accuracy due to the need to calculate the optical flow map. Given the need for detection accuracy in practical applications where the difference in detection time required is less prominent, a comprehensive analysis shows that the dual micro SSD in this thesis shows some advantages in target detection, demonstrating the effectiveness of the improvements to the SSD in this thesis. The resultant AP values of 20 different categories in the VOC dataset for different models of SSD and dual micro SSD are summarized as shown in Figure 7. This thesis focuses on detecting motion pedestrian targets, and the AP values in the table show that the dual micro SSD network has a significant improvement effect in detecting a subset of person target categories, indicating that this improvement is desirable. One of the shortcomings of the performance is that the update of SGD does not follow the correct direction will cause fluctuations in the optimization results, but on the other hand, the fluctuation effect brought by SGD is not necessarily completely unfavorable because it may make the optimization results fluctuate from the current local extreme to another better local extreme or even global extreme.

In the experimental process, the dual micro SSD network model is trained, and the accuracy of the results will be improved with the number of iterations within a reasonable range of learning rate, as shown in Figure 8; in addition, different learning rates will make the accuracy of detection vary with the same number of iterations. In general, the learning rate of bias in SSD network is set to be two times of the learning rate of weight.

Motion target detection and tracking technology involves artificial intelligence, deep learning, and image processing aspects, which have very universal applications in many fields, such as intelligent transportation, medical health, machine assistance, and military aviation. Facing such a promising direction, this thesis focuses on deep learning-based motion target detection and tracking and prediction. Neural network-based target detection and tracking algorithms have received a lot of attention from researchers. In this paper, we design and complete several sets of experiments to improve the SSD network using the VOC dataset containing 20 types of target objects and the filmed video set as the experimental objects of the detection model and conduct a series of comparative analyses and conclusions on the effectiveness of the experimental model using the experimental evaluation metrics. In the target detection study, we combined the current deep learning-based target detection modeling techniques, reviewed a large number of references and rich weblogs, summarized and analyzed the advantages and disadvantages of the current techniques, and selected the SSD neural network as the basis to complete the motion target detection and tracking task in this thesis. The SSD network was first trained using VOC dataset and then applied to the actual shooting scene video, which resulted in false detection, and then the SSD network was improved, and its network structure was modified. The detection and tracking model with the dual-micro kernel phase-to-phase processing mode and the motion target detection and tracking model with this network structure does not have any false detection in the detection of the moving pedestrians in the video and ensures the stability of its detection and tracking.

In order to visualize the SSD network successfully, completing the tracking of the pedestrian target, the trajectories and detections between two consecutive before-and-after frames are connected to form a continuous pedestrian target tracking trajectory. In summary, this thesis model completes the detection and tracking of the moving target and its trajectory prediction. In the process of this trajectory prediction task, this paper compares two prediction methods based on LSTM networks in terms of reliability and correctness of the output results: one is point-by-point prediction, and the other is complete sequence prediction, and finally the point-by-point prediction method is more accurate in the experimental application according to the actual situation.

In this paper, all the rectangular detection frames of the pedestrian are identified and saved to the initialized list in the order of before and after video frames, and then all the masses in the list are connected in the form of a drawing, and finally the tracking trajectory of the pedestrian target is formed. For the motion target detection, this chapter uses the improved SSD network to form a deep learning model called dual micro SSD, which is applied to the VOC dataset to effectively improve the accuracy of the target detection results, while ensuring a considerable speed of detection, which is an improvement compared with other models. The motion target detection and tracking method of this thesis is constructed based on this neural network, and the accuracy and stability of the motion target detection and tracking are ensured by the process of repeated experiments and debugging based on the detection and tracking of motion pedestrians in actual videos. The LSTM network is used to predict the trajectory route of pedestrians, and good prediction results are obtained. The estimated range of the future trend of pedestrians was made in order to provide a modest support for autonomous driving. Later research work is needed to try to think and try to solve some realistic challenges.

## 5. Conclusion

For the motion target detection problem, this paper studies the motion target detection method based on deep learning, and by analyzing the optical flow network and background subtraction network based on deep learning, this paper proposes an optical flow-assisted background subtraction network. The method generates samples for background subtraction network pairs by training the optical flow network to detect partial interframe target motion and then avoids the time consumption of optical flow computation by training a small background subtraction network, which is only needed for detection. Experiments demonstrate that the method can achieve detection effects comparable to manual labeling, solving the dependence of existing background subtraction network-based motion target detection methods on manually labeled target masks and having near real-time target detection performance. For the motion target tracking problem, this paper studies the motion target tracking method based on support vector machine and proposes the tracking method of support vector regression and the corresponding online support vector regression solution method based on the analysis of support vector tracking method and structural support vector tracking method. Experiments show that the proposed support vector regression method can achieve the regression performance of existing offline methods and has obvious speed advantage over existing methods. For the motion target tracking problem, the fusion algorithm of different types of trackers is studied in this paper. In this paper, we propose a tracking method that fuses structural support vector machines and correlation filtering. The method achieves the complementary advantages of structural support vector machines for redetection of occluded targets and correlation filters for scale estimation through a tandem-type fusion structure and an alternating update strategy. Experiments show that the method can effectively resist the drift of target tracking with certain redetection capability, which significantly improves the accuracy and robustness of the tracker.

## Figures and Tables

**Figure 1:** Motion target image acquisition and noise reduction.

**Figure 2:** Network structure for target detection.

**Figure 3:** Illustration of convolution operation.

**Figure 4:** Neural network-based trajectory prediction.

**Figure 5:** FlowNet learning rate.

**Figure 6:** Performance comparison of multiple models on VOC dataset.

**Figure 7:** Detection efficiency improvement of dual SSD.

**Figure 8:** Accuracy versus number of iterations.

## Data Availability

The data used to support the findings of this study are available from the corresponding author upon request.
